This article has been retracted.

# Inhibiting the microglia activation improves the spatial memory and adult neurogenesis in rat hippocampus during 48 h of sleep deprivation

**DOI:** 10.1186/s12974-017-0998-z

**Published:** 2017-11-15

**Authors:** Meetu Wadhwa, Amit Prabhakar, Koushik Ray, Koustav Roy, Punita Kumari, Prabhash Kumar Jha, Krishna Kishore, Sanjeev Kumar, Usha Panjwani

**Affiliations:** 1 Defence Institute of Physiology and Allied Sciences (DIPAS), Defence Research and Development Organization (DRDO), Lucknow Road, Timarpur, Delhi, India; 2 Neurophysiology Division, Defence Institute of Physiology and Allied Sciences (DIPAS), Defence Research and Development Organization (DRDO), Lucknow Road, Timarpur, Delhi, -110 054 India

**Keywords:** Sleep deprivation, Minocycline, Spatial memory, Microglia, Cytokines, Neuroinflammation, Neurogenesis

## Abstract

**Background:**

Sleep deprivation (SD) leads to cognitive impairment. Neuroinflammation could be a significant contributing factor in the same. An increase in regional brain pro-inflammatory cytokines induces cognitive deficits, however, the magnitude of the effect under SD is not apparent. It is plausible that microglia activation could be involved in the SD-induced cognitive impairment by modulation of neuronal cell proliferation, differentiation, and brain-derived neuronal factor (BDNF) level. The present study aimed to evaluate the possible beneficial effect of minocycline in amelioration of spatial memory decline during SD by its anti-inflammatory and neuroprotective actions. We scrutinized the effect of minocycline on the inflammatory cytokine levels associated with glial cells (microglia and astrocytes) activity and neurogenesis markers crucial for behavioral functions during SD.

**Methods:**

Male Sprague-Dawley rats weighing 230–250 g were sleep deprived for 48 h using automated cage shaking apparatus. The spatial memory was tested using MWM apparatus immediately after completion of SD with and without minocycline. The animals were euthanized, blood was collected, and brain was extracted for neuroinflammation and neurogenesis studies. The set of experiments were also conducted with use of temozolomide, a neurogenesis blocker.

**Results:**

Minocycline treatment increased the body weight, food intake, and spatial memory performance which declined during SD. It reduced the pro-inflammatory and increased the anti-inflammatory cytokine levels in hippocampus and plasma and inhibited the reactive gliosis in the hippocampus evidenced by improved cell count, morphology, and immunoreactivity. Additionally, minocycline administration promoted neurogenesis at different stages: proliferation (BrdU, Ki-67), differentiation (DCX) cells and growth factor (BDNF). However, no significant change was observed in maturation (NeuN) during SD. In addition, molecules related to behavior, inflammation, and neurogenesis were shown to be more affected after temozolomide administration during SD, and changes were restored with minocycline treatment. We observed a significant correlation of neurogenesis with microglial activation, cytokine levels, and spatial memory during SD.

**Conclusion:**

The present study demonstrated that the SD-induced decline in spatial memory, neuronal cells proliferation, differentiation, and BDNF level could be attributed to upregulation of neuroinflammatory molecules, and minocycline may be an effective intervention to counteract these changes.

**Graphical abstract:**

Microglial activation is involved in SD-induced changes in inflammatory molecules, neurogenesis, and spatial memory.

**Electronic supplementary material:**

The online version of this article (10.1186/s12974-017-0998-z) contains supplementary material, which is available to authorized users.

## Highlights

Sleep deprivation (SD) impairs spatial memory by suppressing adult hippocampal neurogenesis.

Inflammatory cytokines balance is disturbed via glial cells activation during SD.

Minocycline improved the behavioral, inflammatory, and neurogenesis consequences of SD.

Neuroinflammation is involved in SD-induced changes in neurogenesis and spatial memory.

## Background

Brain and immune system involve a bi-directional communication mechanism, where glial cells, resident immune cells of the brain, hold a vital position [1, 2]. Neuronal and glial cells interact with each other to maintain the brain homeostasis and integrate to promote the neurogenesis and memory processes [3–5]. Normally, glial cells exist in resting state, but under stress or pathological conditions, they become activated and increase the release of the pro-inflammatory molecules causing neuroinflammation that is detrimental to neurogenesis and further impair spatial memory [6, 7].

In addition, glial cells secrete several sleep regulatory substances (SRSs) including multi-functional cytokines [8, 9]. Cytokines are the potent molecules involved in sleep, and also get stimulated during sleep. Despite the growing number of evidence supporting the fact that sleep loss modifies the immune response and affects the level of pro- and anti-inflammatory molecules, leading to cognitive impairment [10–12], the underlying cellular mechanism is still not clearly understood.

Hippocampus is one of the important brain regions that are involved in spatial memory [13–15]. It is likely that neurogenesis mainly occurs in the subventricular zone (SVZ) of lateral ventricles and subgranular zone (SGZ) of dentate gyrus (DG) region of the hippocampus and is responsible for the spatial learning and memory integration. Previous studies showed that sleep promotes hippocampal neurogenesis**-**mediated spatial learning and memory. Simultaneously, the hippocampus is the most vulnerable brain region under stress or other pathological conditions [10, 16–20]. Available reports have shown that both acute and chronic sleep deprivation (SD) cause spatial memory impairment through changes in neurogenesis at different stages (proliferation, survival, differentiation, even maturation) in the hippocampus [21, 22].

A large number of studies have shown that inhibition of microglial cells activation improves the neurogenesis and cognitive performance [23, 24]. In particular, inhibition of microglia activation by minocycline (a broad spectrum antibiotic, anti-inflammatory drug) has a profound neuroprotective effect associated with the improvement of spatial memory and neurogenesis during neuroinflammatory conditions [3, 14, 25]. Therefore, we selected minocycline as a therapeutic approach against the SD-induced neuroinflammation-mediated changes in adult neurogenesis and spatial memory impairment.

We hypothesized that spatial memory impairment during SD with declined adult neurogenesis is mainly due to activated microglia-induced neuroinflammation. The present study aimed to assess the effect of minocycline on the spatial memory, gliosis, and inflammatory cytokine levels during 48 h SD. We also evaluated the impact of minocycline on neuronal cell proliferation, differentiation, maturation, and growth factor during SD and the possible correlation between neurogenesis, spatial memory, cytokines, and microglial cells.

## Methods

### Animal

Adult male Sprague-Dawley rats (230–250 g) were placed in pairs in the plexiglass cage in the institutional animal house, maintained at standard environmental conditions of temperature (25 ± 2 °C) and humidity (55 ± 2% RH). Food pellets (Lipton Pvt. Limited) and water were provided to animals. The experiments were done in consistence with the guidance of Institutional Animal Ethics Committee. All efforts were made to minim ize the number of animals within the statistical limit and pain to animals at each step. Animals were handled regularly by the experimenter and habituated to the experimental conditions to avoid other stress. All experiments were done during the light period of the day.

### Experimental design

The present study was sub-divided into three phases:

#### Standardization of the minocycline dose during SD

Minocycline drug was standardized at three doses (10, 5, and 2 mg/kg) to select the minimum dose producing maximum behavioral and anti-inflammatory outcomes during SD conditions. Following behavioral screening, rats were randomly divided into different groups: cage control with vehicle-treated (CC + Veh); cage control with minocycline (10 mg/kg) treated [CC + Mino (10 mg/kg)]; cage control with minocycline (5 mg/kg) treated [CC + Mino (5 mg/kg)]; cage control with minocycline (2 mg/kg) treated [CC + Mino (2 mg/kg)]; sleep deprived for 48 h with vehicle treated (SD + Veh); sleep deprived for 48 h with minocycline (10 mg/kg) treated [SD + Mino (10 mg/kg)]; sleep deprived for 48 h with minocycline (5 mg/kg) treated [SD + Mino (5 mg/kg)]; sleep deprived for 48 h with minocycline (2 mg/kg) treated [SD + Mino (2 mg/kg)]. Behavioral and inflammatory cytokine profiles were estimated.

#### Evaluation of the interaction between the neuroinflammation, neurogenesis and spatial memory during SD at the standardized dose of minocycline

Rats were randomly divided into different groups after the behavioral screening: cage control with vehicle treated (CC + Veh); cage control with minocycline treatment at the standardized dose (CC + Mino); sleep deprived for 48 h with vehicle treated (SD + Veh); sleep deprived for 48 h with minocycline treatment at the standardized dose (SD + Mino). Glial cells activation and adult neurogenesis along with physiological, behavioral, and inflammatory profile were investigated.

#### Validation of the study

To validate the observations, the effect of temozolomide was observed at behavioral, biochemical as well as cellular level. After the behavioral screening, different groups were assigned: cage control with temozolomide treated (CC + TMZ); cage control with temozolomide and minocycline treated (CC + TMZ + Mino); sleep deprived for 48 h with temozolomide-treated (SD + TMZ); sleep deprived for 48 h with temozolomide and minocycline-treated (SD + TMZ + Mino).

There were minimum five rats in each group. Body weight and food intake were measured every day. Animals underwent SD and drug treatment simultaneously. Further animals were immediately taken for the spatial memory test using Morris water maze (MWM) apparatus. After that rats were immediately euthanized and brains were extracted for further studies. The schematic experimental protocol is shown in the Fig. 1.

**Fig. 1:** Timeline of the experimental design. **a** Minocycline dose standardization. **b** Study design at the selected dose of minocycline. **c** Study validation

### SD procedure

Based on our previously reported observation [26], we selected 48-h SD exposure for this study. Animals were sleep deprived for 48 h continuously in the novel automated cage shaking apparatus developed in our lab as per the protocol of Wadhwa et al. [27]. Animals were placed in the experimental 2 SD cages separately housed in the same environmental conditions as in the animal facility. Food and water were provided to rats. Based on animal’s movement, ANY-maze software tracked the immobility and freezing behavior of an animal with the help of IR camera placed overhead. Whenever the immobility and freezing were found to be 30 and 5 s, respectively, the software predicted the animal as sleeping and immediately sent input signals to the ANY-maze interface and shaking controller simultaneously, which in turn provided the vibration and sound as output to awaken the animal.

### Drug administration

Minocycline Hydrochloride (Sigma-Aldrich, USA), dissolved in normal saline, was administered to the rats daily by intraperitoneal (i.p.) route, once a day in the morning time, during 48 h of SD. Minocycline at 10, 5, and 2 mg/kg body weight were used to standardize the dose on the behavioral and biochemical scale. The minimum dose of minocycline showing maximum effect was selected, and it was in accordance with some previous studies [28–30].

### Temozolomide (TMZ) administration

Temozolomide, an alkylating/anti-proliferating agent, has been used as a neurogenesis inhibitor [31]. Temozolomide (Sigma-Aldrich, USA, 25 mg/kg in normal saline, i.p.) was given to rats daily during 48 h of SD. The dose of temozolomide was selected based on previous studies [32, 33].

### BrdU labeling

BrdU (5-bromo-2′-deoxyuridine), a thymidine analog, is used for marking the proliferating cells [16]. BrdU was dissolved in the sterile physiological saline solution containing 0.007 N sodium hydroxide. BrdU at 50 mg/kg body weight dose was given to rats intraperitoneally.

### Body weight and food intake measurements

We measured the body weight and food intake of the rats at regular intervals before experiments. Throughout the study, a constant amount (150 g) of food pellets was provided to rats in the control cage as well as in SD chamber. Body weight and food intake were measured every day in the morning.

### Spatial memory test

Spatial memory is a navigational memory depending on the spatial orientation and generally tested using MWM test procedure. The environmental conditions (temperature, humidity, light, and sound) were properly maintained, and the test was performed as per the protocol of Chauhan et al. [34]. The test apparatus comprised of a black painted circular pool (210 cm diameter and 53 cm height), and a transparent platform. The pool was filled with clean water a little over the platform and maintained at a temperature of 25 ± 2 °C. A camera was placed overhead the water pool and was attached to the ANY-maze software (Stoelting, USA) for assessment.

The testing paradigm consisted of mainly four phases: habituation, training, probe test, and test phase. In the habituation phase, the rats were subjected to the water pool without a platform for 5 min and allowed to swim. Behaviorally and physically healthy rats without having any stereotypic characteristics were selected for further study to minimize the effect of the stress. In the training phase, the MWM apparatus was equally divided into four zones (Z1, Z2, Z3, Z4) and the platform was placed in the Z4 zone, which was denoted as ISLAND zone. Rats were placed into Z1, Z2, Z3, and Z4 zones sequentially for 60 s facing the animal head on the wall side of the pool and allowed to search the platform. If the rat failed to find the platform within 1 min, the experimenter guided the rat to the platform and allowed to sit on the platform for 15 s. After that, the rat was taken out of the pool and dried with a towel and placed back to the home cage. Likewise, rats received four trials per day with an inter-trial interval of 5 min. The training session was 7 days (TD1-TD7). After completion of training or before subjecting the animals to SD (eighth day), the rats were tested by subjecting them to the Z2 zone (opposite to ISLAND zone) for 1 min and were allowed to find the platform to confirm whether they were adequately trained or not (probe test). If the animals succeeded to locate the platform within 10 s, it meant that the animals were well trained and ready for subjecting to SD. After completion of 48 h of SD, rats immediately underwent the test phase (with hidden platform and without hidden platform) in which they were again placed in the opposite to ISLAND zone, i.e., Z2 zone for 1 min. Different parameters such as latency, path length, path efficiency to reach the platform (with the hidden platform), and number of entries, time spent in the ISLAND zone (without hidden platform) were evaluated under probe and spatial memory test.

### Blood, tissue collection, and processing

Immediately after the behavioral test, rats were given the anesthetic dose of ketamine 80 mg/kg-xylazine 20 mg/kg. Blood was collected from the left ventricle and centrifuged at 3500 rpm for 15 min, plasma was separated, aliquoted, and stored at − 80 °C for further analysis.

For hippocampus collection, the whole brain was extracted after anesthetizing the rats by giving ketamine 80 mg/kg-xylazine 20 mg/kg in combination. The hippocampus region was isolated from the whole brain kept on ice, washed with 0.1 M phosphate-buffered saline (PBS) solution and stored at − 80 °C. Hippocampal tissue was homogenized in 1× PBS solution containing protease inhibitor cocktail using with the help of polytron homogenizer and centrifuged at 10,000 rpm for 15 min at 4 °C. The supernatant was separated carefully and stored at − 80 °C for enzyme-linked immunosorbent assay (ELISA).

### Inflammatory gene expression assay

The total RNA was isolated from hippocampal tissue using TRIZOL reagent (Sigma) according to the previously described protocol [35]. After quantitative determination of RNA using a Nanodrop (Thermo Fisher Scientific, USA) that measured absorbance at 260 and 280 nm. The integrity and size distribution of total purified RNA was checked by denaturing agarose gel electrophoresis and ethidium bromide staining. Agarose gel (1%) was prepared in TBE (Tris-Borate EDTA) for this purpose. RNA was reverse-transcribed to cDNA using an RT2 first strand cDNA Synthesis Kit (QIAGEN Sciences, Maryland, USA), according to the manufacturer’s instruction. Relative quantitative analysis of the gene expression of interleukins and tumor necrosis factor for each group was done by employing RT^2^ Profiler inflammatory cytokines and receptor array (QIAGEN Sciences, Maryland, USA) using RT^2^ SYBR® Green qPCR master mix (QIAGEN Sciences, Maryland, USA). The gene expression analysis was done using software available online at www.sabiosciences.com, after normalization of each gene (Ct) to the housekeeping genes.

### Estimation of cytokine levels in collected plasma and hippocampal tissue

We measured the cytokine (IL-6, TNF-α, IL-4, IL-10, and IL-1β) levels in plasma and hippocampal lysates by using their respective ELISA kits, procured from BD Biosciences and R&D Systems, Minneapolis, MN, USA. The assay was performed according to the prescribed manufacturer’s protocol.

### Immunohistochemistry (IHC)

Immunohistochemical analysis mainly consists of the following stages: whole brain collection, sectioning and immunolabeling. Rats were first transcardially perfused with ice chilled 0.1 M PBS solution (1×), later with ice chilled 4% paraformaldehyde (PFA) solution prepared in 1× PBS solution after anesthetizing the rats with urethane (1.2 g/kg, i.p.) prepared in normal saline. The whole brain was extracted and stored in 4% PFA at 4 °C (brain collection). Brains were sequentially placed in the different grades of sucrose solution (10, 20, and 30%) prepared in 1× PBS until they sank to the bottom. Coronal sections of the hippocampus (30 μm thickness) were collected in 0.02% sodium azide solution (anti-fungal agent) using cryostat instruments (Leica Pvt. Limited) (sectioning).

The immunolabeling protocol for all the antibodies was same except for BrdU and Iba-1 proteins. For BrdU immunostaining, DNA denaturation is required before immunolabeling, for which sections were pre-treated with 2 M hydrochloride and Triton-X 100 at 37 °C for 45 min followed by 10 min washing in borate buffer (pH 8.5). Sections were then labeled with rat anti-BrdU antibody (1:250, Abcam, Cambridge, USA) at 4 °C for 40 h.

Similarly, for Iba-1 immunolabeling membrane permeabilization was done before the step of blocking. The sections were incubated with 0.25% Triton-X 100 for 30 min at room temperature and were washed with IHC buffer (2–3 times). The IHC buffer used for Iba-1 labeling was 0.1 M PBS solution containing Triton-X 100. Bovine serum albumin (BSA, 2–3%) was used as a blocking buffer. Sections were incubated with Goat anti-Iba-1 primary antibody (1:250, Sigma-Aldrich, USA) prepared in 1.5% BSA solution at 4 °C for 40 h.

Dorso-ventral hippocampal sections were taken and washed with IHC buffer (0.1 M PBS solution containing Tween-20). Antigen retrieval was done in the sodium citrate buffer (pH 6.0) in boiling water bath for 10 min. Sections were then appropriately washed at room temperature in the IHC buffer. Subsequently, sections were then blocked with 10% normal goat solution (NGS) in PBS containing 0.03% Triton-X 100 for 2 h at room temperature. Immunolabeling was done by incubating the sections with specific antibodies; rabbit anti-GFAP (1:500, Abcam, Cambridge, USA), rabbit anti-DCX (1:500, Abcam, Cambridge, USA), rabbit anti-NeuN (1:500, Abcam, Cambridge, USA) and rabbit anti-BDNF (1:500, Abcam, Cambridge, USA), freshly prepared in blocking buffer, at 4 °C for 40 h. Sections were then washed with IHC buffer (3–4 times) at 5 min interval. Endogenous peroxidase activity was blocked by incubating the sections with 0.3% hydrogen peroxide (H_2_O_2_) solution with subsequent washing with IHC buffer. Thereafter, sections were incubated with the horseradish peroxidase (HRP) conjugated specific secondary antibodies: Goat anti-Rt (1:500, Abcam, Cambridge, USA), Horse anti-Goat (1:500, Sigma-Aldrich, USA), respectively, at room temperature for 2 h. Sections development was done in 3,3′-diaminobenzidine (DAB) tetrahydrochloride and hydrogen peroxide (H_2_O_2_) solution prepared in PBS with subsequent washing. Sections underwent dehydration process using a graded solution of ethanol (50%, 70%, 90% and absolute alcohol) and xylene treatment after transferring to the gelatine-coated slide and dried. Finally, the sections were DPX mounted and allowed to dry at room temperature. Negative control lacking primary antibody was taken simultaneously for accuracy (immunolabeling).

### Image acquisition and analysis

Sections were visualized under bright field microscope (Olympus, Melville, NY, BX51TF) using ×10, ×20 and ×40 objective lens, and the images were taken by the inbuilt camera of the microscope. The preparation of images in representable form (tiff format) and measurement of immunoreactivity of proteins were done using GIMP, and ImageJ software. Stereoinvestigator software was used for the cell counting, and the morphology of microglial cells (Iba-1) and astrocytes (GFAP) was assessed by sholl analysis.

### Statistical analysis

Statistical analysis was done using GraphPad Prism software, San Diego, California, USA. Data were analyzed using Student’s *t* test, one-way ANOVA followed by a post hoc test (parametric and non-parametric) as per applicability. Values were expressed as mean ± SEM. The value of *p* < 0.05 was considered to be statistically significant. Mean percentage of control value was used for graphical representation.

## Results

### Sleep deprivation promotes gliosis and thus impairs spatial memory

We foremost evaluated the effect of SD on spatial memory in rats. We observed significantly increased latency (Fig. 2a) and path length (Fig. 2b) with reduced path efficiency (Fig. 2c) to reach the platform following 48 h of SD. The reduced number of entries (Fig. 2d) and time spent (Fig. 2ein the ISLAND zone were also observed in sleep-deprived rats. Prior to the spatial memory test, all the animals underwent habituation, 7 days training phase [TD1-TD7] (Additional file 1: Figure S1A–D) followed by probe test with (Additional file 1: Fig. S1E–G) and without (Additional file 1: Figure S1H, I) platform.

**Fig. 2:** Sleep deprivation induces changes in spatial memory, cytokine levels and glial cells immunoreactivity in rats. Behavioral study parameters. **a** Latency. **b** Path length. **c** Path efficiency. **d** Number of entries. **e** Time spent. Immunoreactivity of **f** GFAP. **g** Iba-1 in DG, CA1, and CA3 region of the hippocampus. Fold changes in the **h** pro-inflammatory cytokines. **i** Anti-inflammatory cytokines in the hippocampus. *p < 0.05 when compared to control treated with vehicle. Parametric and non-parametric Student *t* test was applied for the test parameters as required

Investigation of glial cells indicated the enhanced GFAP (Fig. 2f) and Iba-1 (Fig. 2g) immunoreactivity in DG, CA1, and CA3 region of the hippocampus, suggesting the involvement of neuroinflammation in SD-induced spatial memory impairment. Thus, next, we measured the concentration of inflammatory cytokines in the hippocampus of SD rats. A significant upsurge in pro-inflammatory, TNF-α, IL-1β, and IL-6 with subsequently declined concentration of anti-inflammatory, IL-4, and IL-10 (Fig. 2h, i), molecules were observed during 48 h of SD. We also found a significant reduction in body weight (Additional file 1: Figure S1J) and food intake (Additional file 1: Figure S1K) in SD rats. These results suggest that SD stimulates glial cells activation resulting in the release of pro-inflammatory cytokines and spatial memory impairment.

### Evidence for inflection of inflammatory responses during SD leading to spatial memory impairment

The observed results that neuroinflammation hastens spatial memory impairment during SD urged to scrutinize the extent of the release of inflammatory cytokines from the activated glial cells. We first established the smallest effective dose of minocycline treatment against SD and associated consequences. A total of three doses (10, 5, and 2 mg/kg) were administered in both control and SD groups. Minocycline treatment with 5 mg/kg dose was found to be significantly effective against SD in majority of the tests such as body weight, food intake (Additional file 2: Figure S2A), spatial memory tests (Additional file 2: Figure S2B–F), pro- (Additional file 2: Fig. S2G–I) and anti-inflammatory cytokine levels (Additional file 2: Figure S2J, K) in plasma, hence, considered for further experiments with minocycline treatment.

We performed the MWM-based spatial memory test during SD with minocycline. Rats underwent training (Additional file 3: Figure S3A–C) and probe test (Additional file 3: Figure S3D–H) before the spatial memory test. We recorded the track plot (Fig. 3a) for all the four groups. A considerable reversal of spatial memory was observed post minocycline treatment to SD rats. A significantly improved performance as reduced latency (Fig. 3c) and path length (Fig. 3d) with enhanced path efficacy (Fig. 3e) to reach the platform was observed. Track plot recording without platform (Fig. 3b) shown spatial memory improvement after minocycline administration during SD, confirmed by an increased number of entries (Fig. 3f) and time spent (Fig. 3g) in the ISLAND zone.

Next, we looked for the functional involvement of inflammatory responses in altered behavioral changes. We studied the concentration of well documented inflammatory cytokines and observed significant increase in the levels of pro-inflammatory: TNF-α (Fig. 4a), IL-1β (Fig. 4b) and IL-6 (Fig. 4c) with decreased anti-inflammatory cytokines: IL-4 (Fig. 4d) and IL-10 (Fig. 4e) during 48 h SD in hippocampus and plasma (Additional file 3: Figure S3I–M).

Furthermore, our real-time PCR results for these inflammatory response genes confirmed the expression pattern of TNF-α (Fig. 4f), IL-1β (Fig. 4g), IL-6 (Fig. 4h), IL-4 (Fig. 4i), and IL-10 (Fig. 4j) after SD and further improved towards basal values by minocycline treatment. Figure 4k presents the heat map for the expression of inflammatory cytokines. The expression pattern of these molecules was found similar in both hippocampus and plasma (Fig. 4l).

**Fig. 3:** Minocycline treatment improves the spatial memory performance following SD. Track plot of the performance of rats. **a** With platform. **b** Without platform. Study parameters. **c** Latency. **d** Path length. **e** Path efficiency [with hidden platform]. **f** Number of entries. **g** Time spent [no platform]. *p < 0.05 when compared to control treated with vehicle. ^ϕ^ *p* < 0.05 when compared to sleep deprived treated with vehicle. One-way ANOVA with Bonferroni post hoc test was applied for latency, path length to reach the platform, time spent in the target zone, and Kruskal-Wallis with Dunn’s post hoc test for path efficiency to reach the platform, number of entries in the ISLAND zone

**Fig. 4:** Minocycline treatment balances the fold changes in the inflammatory cytokines in hippocampus during SD. Fold changes in the inflammatory cytokines in the hippocampus at protein level. **a** TNF-α. **b** IL-1β. **c** IL-6. **d** IL-4. **e** IL-10. Fold changes in the inflammatory cytokines in the hippocampus at mRNA level. **f** TNF-α. **g** IL-1β. **h** IL-6. **i** IL-4. **j** IL-10. **k** Heat map showing the pro- and anti-inflammatory cytokines in hippocampus and plasma. **l** Pro/anti-inflammatory cytokines ratio in the hippocampus and plasma. *p < 0.05 when compared to control treated with vehicle, ^ϕ^ *p* < 0.05 when compared to sleep deprived treated with vehicle. One-way ANOVA with Bonferroni post hoc test was used

### Immunohistochemical analysis commends SD-induced gliosis mediated neuroinflammation

To scrutinize the relation between inflammation and glial cells activation, we first analyzed the immunoreactivity of astrocytes and microglial cells activation markers during SD. Figure 5a presents the astrocyte expression of GFAP in DG, CA1, and CA3 regions. We had not observed significantly increased GFAP immunoreactivity in DG (Fig. 5b), CA1 (Fig. 5c), and CA3 (Fig. 5d) region during SD and following minocycline treatment as well. Additionally, we observed increased microglial cell expression during SD (Fig. 5e). Minocycline, a microglia activation inhibitor, effectively decreased the immunoreactivity of Iba-1 during 48 h SD in DG (Fig. 5f), CA1 (Fig. 5g), and CA3 (Fig. 5h) region of the hippocampus.

**Fig. 5:** Minocycline inhibits the glial cells immunoreactivity in rat hippocampus following SD. **a** Representable image of astrocytes expression in DG, CA1, and CA3 regions of the hippocampus. GFAP immunoreactivity quantification in **b** DG region. **c** CA1 region. **d** CA3 region of the hippocampus. **e** Representable image of microglial cells expression in DG, CA1, and CA3 regions of the hippocampus. Iba-1 cell immunoreactivity quantification in **f** DG region. **g** CA1 region. **h** CA3 region of the hippocampus. *p < 0.05 when compared to control treated with vehicle. ^ϕ^ *p* < 0.05 when compared to sleep deprived treated with vehicle. One-way ANOVA with Bonferroni post hoc test was used

Further, we verified morphological alterations in the glial cells. Different stages of the astrocyte (resting, activated) and the microglial cell (resting, intermediate, activated) were presented as intersectional and segmented images in Fig. 6a, b, respectively. Exposure to 48 h SD significantly altered the morphology of astrocytes and microglia respectively as increased soma density (Fig. 6c, i) and soma area (Fig. 6d, j) with decreased sum inters (Fig. 6e, k), mean inters (Fig. 6f, l), ramification index (Fig. 6g, m), and glial length (Fig. 6h, n). We observed remarkable improvement in glia cells morphology after minocycline treatment during SD.

Next, we performed the cell counting analysis of resting, intermediate, and activated stage microglial cells. Iba-1 positive cell count was significantly decreased at resting stage in DG and CA3 region after 48 h SD, whereas, extensively increased count was observed at an activated stage in all the three DG, CA1, and CA3 regions (Fig. 6o–q). Additionally, changes in total microglial cell count were not significant in DG, CA1, and CA3 regions (Fig. 6r–t). However, administration of minocycline considerably improved the cell count altered after SD. These observations confirmed the involvement of gliosis in SD-mediated consequences that get improved with the treatment of minocycline.

**Fig. 6:** Minocycline improves SD-induced alteration in the glia cells morphology and cell count in rat hippocampus. Representable image (intersection and segmented mask) of **a** normal and activated astrocyte. **b** Resting, intermediate, and activated stage microglial cell. Changes in the **c** soma density. **d** Soma area. **e** Sum inters. **f** Mean inters. **g** Ramification index. **h** Astrocyte length of astrocyte in DG, CA1, and CA3 regions of the hippocampus. Changes in the **i** soma density. **j** Soma area. **k** Sum inters. **l** Mean inters. **m** Ramification index. **n** Microglial length of microglia in DG, CA1, and CA3 regions of the hippocampus. Changes in the microglial cell count at different stages (resting, intermediate, and activated) in **o** DG region. **p** CA1 region. **q** CA3 region of the hippocampus. Total microglia cell count in **r** DG region. **s** CA1 region. **t** CA3 region of the hippocampus.*p < 0.05 when compared to control treated with vehicle. ^ϕ^ *p* < 0.05 when compared to sleep deprived treated with vehicle. One-way ANOVA with Bonferroni post hoc test was used for the analysis of soma density, soma area, astrocyte length, and microglia size while Kruskal-Wallis with Dunn’s post hoc test was applied for sum inters, mean inters, ramification index parameters, and cell count analysis

### Involvement of neuroinflammation in adult neurogenesis decline during SD

We next examined the neurogenesis that was supposed to be impaired due to neuroinflammation during SD. Figure 7a represents the DG region of the hippocampus. We evaluated the proliferating stage of neurogenesis using Ki-67 (Fig. 7b) and BrdU (Fig. 7c) markers. Reduction in proliferation was observed in SD animals that get improved on minocycline administration as indicated by an increased number of Ki-67 (Fig. 7d) and BrdU (Fig. 7e) positive cells in DG region. Further, we investigated the differentiating cells at proliferating, intermediate and post-mitotic phases in the DG region of the hippocampus (Fig. 7f). We observed potent changes in the expression of doublecortin (DCX), a marker of differentiation, in the DG region during SD (Fig. 7g). A significant decrease in the numbers of DCX positive cells in proliferative, intermediate and post-mitotic phases of differentiation was observed during SD, and the improvement in cells counting post minocycline treatment confirmed the role of inflammation in the decrement of neurogenesis (Fig. 7h). Next, we tend to evaluate whether SD modulates the neurogenesis by altering the expression of NeuN protein during maturation stage in DG region. Nevertheless, we did not observe potent changes in relative mean pixel intensity of NeuN protein (Fig. 7i, j).

We investigated the expression of brain-derived neuronal factor (BDNF) in DG, CA1, and CA3 regions of the hippocampus (Fig. 7k). A prominent decrease in the mean pixel density of BDNF protein in DG, CA1, and CA3 (Fig. 7l) regions was seen which tends to basal value after minocycline treatment. These results suggested that inflammation was promptly involved in neurogenesis decline during SD.

**Fig. 7:** Minocycline treatment improves the proliferating, differentiation, maturating, and growth factor proteins following SD. **a** Identification of the DG region of the hippocampus. Representable image of **b** Ki-67. **c** BrdU cells in DG region of the hippocampus. Changes in the cell count of the **d** Ki-67. **e** BrdU cells in DG region of the hippocampus. Representable image showing **f** different stages of DCX positive cells in the DG region of hippocampus. **g** DCX expression among different groups in the DG region of the hippocampus. **h** Changes in the cell counts of DCX cells in the DG region of the hippocampus at proliferative, intermediate, and post-mitotic stage. **i** Representable image showing NeuN expression in the DG region of the hippocampus. **j** Changes in the relative mean pixel intensity of NeuN in the DG region of the hippocampus. **k** Representable image of BDNF expression in DG, CA1, and CA3 region of the hippocampus. **l** Changes in the relative mean pixel intensity of BDNF protein in the DG, CA1, CA3 region of the hippocampus. *p < 0.05 when compared to control treated with vehicle. ^ϕ^ *p* < 0.05 when compared to sleep deprived treated with vehicle. Kruskal-Wallis with Dunn’s post hoc test was applied for statistical analysis of BrdU, Ki-67, and DCX cell count. One-way ANOVA with Bonferroni post hoc test was used for statistical analysis of NeuN and BDNF protein

### Neurogenesis blockade potentiates the SD-induced neuroinflammation and spatial memory impairment

To establish whether the activation of microglial cells played a causal role in the elevated levels of inflammatory molecules and thus impaired neurogenesis during 48 h SD, we used temozolomide (TMZ, a neurogenesis blocker) with minocycline (a microglia activation inhibitor). Subsequently, we performed a spatial memory test, checked expression levels of inflammatory cytokine, studied gliosis and neurogenesis under SD conditions.

All the experiments were performed in four groups discussed earlier in the method section, and SD of 48 h was considered for all the experiments.

#### Spatial memory test

All the animals underwent training session and probe test (Additional file 4: Figure S4A–I). Figure 8a presents the track plot for spatial memory test with the hidden platform. Combinatorial of SD and temozolomide significantly enhances latency (Fig. 8b), path length (Fig. 8c) and decreased path efficiency (Fig. 8d) to reach the platform. Further, spatial memory test without platform was also performed (Fig. 8e). There was a notable decline in the number of entries (Fig. 8f) and time spent (Fig. 8g) in the ISLAND zone in SD + TMZ group. We observed that minocycline treatment with temozolomide either in the control or SD groups comprehensively improved the altered spatial memory (Fig. 8a–g).

**Fig. 8:** Minocycline improves temozolomide induced spatial memory decline and inflammatory cytokine levels in hippocampus during SD. **a** Track plot of memory test session and study parameters such as **b** latency. **c** Path length. **d** Path efficiency [with hidden platform]. **e** Track plot of memory test session and study parameters such as **f** number of entries. **g** Time spent [no hidden platform]. Fold changes in the inflammatory cytokines in the hippocampus. **h** TNF-α. **i** IL-1β. **j** IL-6. **k** IL-4. **l** IL-10. ^α^ *p* < 0.05 when sleep deprived treated with TMZ compared to control treated with TMZ. ^β^ *p* < 0.05 when sleep deprived treated with TMZ and minocycline compared to sleep deprived treated with TMZ. One-way ANOVA with Bonferroni post hoc test was applied for latency, path length to reach the platform, time spent in the target zone, cytokine levels, and Kruskal-Wallis with Dunn’s post hoc test for path efficiency to reach the platform, number of entries in the target zone

#### Inflammatory cytokines

Significantly increased expression of pro-inflammatory cytokines TNF-α (Fig. 8h), IL-1β (Fig. 8i), IL-6 (Fig. 8j) with decreased levels of an anti-inflammatory cytokine such as IL-4 (Fig. 8k) and IL-10 (Fig. 8l) in the hippocampus of SD + TMZ group rats was observed. However, we found significantly decreased pro-inflammatory and increased anti-inflammatory in both CC + TMZ + Mino and SD + TMZ + Mino groups that suggested the role of minocycline in the amelioration of spatial memory impairment due to inflammatory consequences occurred by the combinational effects of SD and TMZ. Subsequently, we observed similar outcomes when the expression levels of inflammatory cytokine were analyzed in plasma (Additional file 4: Figure S4J–N).

#### Inhibition of hippocampal gliosis by minocycline treatment post-TMZ administration during SD

Next we tried to investigate whether blockade of neurogenesis aggravated gliosis-mediated neuroinflammation during SD and tested the potential contribution of minocycline in improving glial functional health. TMZ administration resulted in visible changes in astrocytes (Fig. 9a) and microglial cells (Fig. 9e) expression in SD + TMZ group. We observed minocycline significantly reduced the GFAP (Fig. 9b–d) and Iba-1 immunoreactivity (Fig. 9f–h) in DG, CA1, and CA3 regions of hippocampus respectively that were altered due to the TMZ administered during SD. Furthermore, we also observed improvement in the morphological alterations in astrocytes and microglia bent by TMZ administration along with SD. Minocycline significantly reduced soma density (Fig. 10a), soma area (Fig. 10b), sum inters (Fig. 10c) with enhanced mean inters (Fig. 10d), ramification index (Fig. 10e), and astrocyte length (Fig. 10f) in the astrocytes altered by TMZ administration. Similar outcomes were observed for microglia morphology analysis (Fig. 10g–l).

Additionally, we observed significant normalization of Iba-1 positive cell counts by minocycline treatment at the resting, intermediate, and activated stages of DG (Fig. 10m), CA1 (Fig. 10n), and CA3 (Fig. 10o) regions of the hippocampus. Total microglial cell count was also found to be significantly reduced in SD + TMZ + Mino group relative to SD + TMZ group (Fig. 10p–r).

**Fig. 9:** Minocycline inhibited the temozolomide induced changes in glial cell immunoreactivity in rat hippocampus following SD. **a** Representable image of astrocyte expression in DG, CA1, and CA3 regions of the hippocampus. GFAP immunoreactivity quantification in **b** DG region. **c** CA1 region. **d** CA3 region of the hippocampus. **e** Representable image of microglial cells expression in DG, CA1, and CA3 regions of the hippocampus. Iba-1 cell immunoreactivity quantification in **f** DG region. **g** CA1 region. **h** CA3 region of the hippocampus. ^α^ *p* < 0.05 when sleep deprived treated with TMZ compared to control treated with TMZ. ^β^ *p* < 0.05 when sleep deprived treated with TMZ and minocycline compared to sleep deprived treated with TMZ. One-way ANOVA with Bonferroni post hoc test was used for statistical analysis

**Fig. 10:** Minocycline improves glia cells morphology and cells count in hippocampus following temozolomide administration during SD. Changes in the **a** soma density. **b** Soma area. **c** Sum inters. **d** Mean inters. **e** Ramification index. **f** Astrocyte length of astrocyte in DG, CA1, and CA3 regions of the hippocampus. Changes in the **g** soma density. **h** Soma area. **i** Sum inters. **j** mean inters. **k** Ramification index. **l** Microglial length of microglia in DG, CA1, and CA3 regions of the hippocampus. Changes in the microglial cell count at different stages (resting, intermediate, and activated) in **m** DG region. **n** CA1 region. **o** CA3 region of the hippocampus. Total microglia cell count in **p** DG region. **q** CA1 region. **r** CA3 region of the hippocampus. ^α^ *p* < 0.05 when sleep deprived treated with TMZ compared to control treated with TMZ. ^β^ *p* < 0.05 when sleep deprived treated with TMZ and minocycline compared to sleep deprived treated with TMZ. One-way ANOVA with Bonferroni post hoc test was used for the analysis of soma density, soma area, astrocyte length, and microglia size while Kruskal-Wallis with Dunn’s post hoc test was applied for sum inters, mean inters, ramification index parameters, and cell count analysis

#### Minocycline stabilizes the TMZ-induced alteration in adult neurogenesis

Subsequently, we observed prominent proliferation indicated by the improved number of Ki-67 (Fig. 11a) and BrdU (Fig. 11b) positive cells in DG region on minocycline treatment relative to SD + TMZ group. Figure 11c presented expression of DCX positive cells as differentiation marker. Minocycline efficiently increased the number of DCX positive cells at all three (proliferative, intermediate, and post-mitotic) stages (Fig. 11d). It also improved the maturation phase of neurogenesis as increased mean pixel intensity of NeuN was observed in SD + TMZ + Mino group (Fig. 11e, f). Last, we looked for expression of growth factor in the presence of TMZ with or without minocycline (Fig. 11g) and observed a significant reversal in BDNF mean pixel intensity in DG (Fig. 11h), CA1 (Fig. 11i), and CA3 (Fig. 11j) regions with respect to SD + TMZ group. These data evidenced the effectiveness of minocycline in the improvement of the gliosis, neuroinflammation, and spatial memory impairment.

**Fig. 11:** Minocycline treatment improves the temozolomide induced alteration of the neurogenesis proteins during SD. Changes in the cell counts of the **a** Ki-67. **b** BrdU cells in DG region of the hippocampus. **c** Representable image displaying the changes in DCX expression. **d** Cell counts of DCX cells in the DG region of the hippocampus at proliferative stage, intermediate stage, and post-mitotic stage. **e** Changes in the NeuN expression in the DG region. **f** Relative mean pixel intensity of NeuN protein in the DG region of the hippocampus. **g** Representable image of the changes in the BDNF expression in DG, CA1, and CA3 region of the hippocampus. Changes in the relative mean pixel intensity of BDNF protein in the **h** DG. **i** CA1. **j** CA3 region of the hippocampus. ^α^ *p* < 0.05 when sleep deprived treated with TMZ compared to control treated with TMZ. ^β^ *p* < 0.05 when sleep deprived treated with TMZ and minocycline compared to sleep deprived treated with TMZ. Kruskal-Wallis with Dunn’s post hoc test was applied for statistical analysis of cell count. One-way ANOVA with Bonferroni post hoc test was used for statistical analysis of relative mean pixel intensity of NeuN and BDNF proteins

### Neuroinflammation (activated glial cells and altered cytokines expression) underlies in root of SD-induced deterioration of neurogenesis and spatial memory impairment

To investigate the possible strong association as causative behind the proposed SD-mediated changes in spatial memory, inflammatory, and neurogenesis molecules, we evaluated the interrelation of neurogenesis with spatial memory (Fig. 12a), inflammatory cytokines (TNF-α and IL-1β) released from activated microglia (Fig. 12b, c) and activated microglial cells strength (Fig. 12d) under SD stress. We observed a strong negative correlation of BDNF expression, BrdU positive cells count and proliferative DCX cells in the DG region with these mentioned parameters. These results suggested that SD resulted in an increased number of activated microglial cells; tend to enhance the release of pro-inflammatory cytokines. The enhanced levels of cytokines represented neuroinflammation that in turn deteriorated the adult neurogenesis and hampered the spatial memory performance in sleep-deprived rats.

**Fig. 12:** Correlation analysis predicting the interaction between spatial memory, cytokines, activated microglia, and neurogenesis during SD. **a** Adult neurogenesis and spatial memory interaction as shown by correlating latency to reach the platform with the number of BrdU-positive cells, proliferative DCX positive cells, and relative mean pixel intensity of BDNF protein. Interaction between the adult neurogenesis and pro-inflammatory cytokines level as shown by correlation between **b** TNF-α level in hippocampus and the number of BrdU-positive cells, proliferative DCX positive cells, and relative mean pixel intensity of BDNF protein. **c** IL-1β level in hippocampus and the number of BrdU-positive cells, proliferative DCX positive cells, and the relative mean pixel intensity of BDNF protein. Finally, the interaction between neurogenesis and activated microglial cells as shown by **d** correlation of activated microglial cells count in the hippocampus with the number of BrdU-positive cells, proliferative DCX positive cells, and relative mean pixel intensity of BDNF protein

## Discussion

It has been known that loss of sleep has a detrimental impact on cognitive functions [10]. Microglia activation, a key factor in neuroinflammation is inhibited by minocycline in various inflammation-related disease conditions like Alzheimer’s disease, multiple sclerosis, and ischemic stroke [7, 36]. An improvement in spatial memory by minocycline, by a reduction in hippocampal neuroinflammation, is in agreement with earlier studies on social deficits [37], colchicine [38], and LPS [39]. The activation of microglia culminates in the release of inflammatory cytokines, enhanced neuroinflammation, and cognitive impairment during stress and other pathological conditions [11, 36, 40–42].

The present study revealed a role of neuroinflammation through microglia activation in the suppression of adult neuronal cell proliferation and spatial memory decline during SD. Inhibition of the microglia activation by minocycline improved the spatial memory and adult neuronal cell proliferation possibly through the upregulation of hippocampal BDNF level during SD. Subsequently, these findings were validated by blocking the neurogenesis and observing the above consequences of SD.

Sleep deprivation activated the glial cells, which increased the release of inflammatory molecules, leading to spatial memory decline. Glial cells activation was evidenced by increased microglial reactivity and deviation from normal microglial morphology along the changes in cell body, branching index and the cell counting ratio of resting and activated microglial cells during SD, this is in agreement with earlier reports on efficacy of minocycline against stress-induced gliosis [2, 39, 41, 43]. Interestingly, we found a non-significant increase in astrocyte immunoreactivity. However, the morphology of astrocytes was significantly altered, indicating astrocytes hypertrophy during SD.

Glial cells activation induced neuroinflammation suppressed the adult neurogenesis in DG which is the hallmark of neurodegenerative diseases [7, 23, 26, 44, 45]. Mueller et al. [46] had reported the involvement of IL-1β signaling in the SD-mediated alterations in cell proliferation. Therefore, we evaluated the relationship of neuroinflammation with neurogenesis on the basis of the microglial activity and cytokine levels during SD. We observed improvement in neurogenesis at proliferation and differentiation stages after minocycline treatment during 48 h of SD along with the improved BDNF level supporting the role of BDNF in sleep regulation and facilitating the neurogenesis [10, 13, 39, 47]. These data point towards the possibility of neuroinflammation as a link between SD-induced adult neurogenesis declines and spatial memory impairment.

In order to validate the role of neuroinflammation in SD-induced impairment in spatial memory and suppression of adult neuronal cell proliferation, temozolomide was used. This led to spatial memory impairment along with extensive glial cells activation and induction of neuroinflammation. We observed decreased body weight, food intake along with the impairment of spatial navigational memory and significantly enhanced pro-inflammatory cytokines concentration that support the earlier findings in other stresses [31–33, 48]. The extensive alteration in the level of inflammatory cytokines (pro and anti) in SD + TMZ group relative to SD + Veh group points to the role of neuronal cells proliferation in disturbance of the pro- and anti-inflammatory cytokines balance leads to memory impairment during SD. These findings were further supported by extensively activated glial cells (astrocytes and microglia) in the form of reactivity, morphology, and cell counts post temozolomide treatment during SD.

Administration of temozolomide potentiated the changes in adult neurogenesis at proliferating, differentiating, and mature neuronal stage with altered growth factor in SD + TMZ group. However, minocycline treatment potentially improved the alterations caused so far due to SD stress with neurogenesis blockade. The negative correlation of neurogenesis with activated microglial cells, pro-inflammatory cytokines, and spatial memory test parameter (Fig. 12) is suggestive to the involvement of SD-induced neuroinflammation in spatial memory impairment and modulating neuronal cells proliferation, and minocycline is an effective intervention in counteracting these changes.

## Conclusions

In conclusion, the present study demonstrated for the first time the role of neuroinflammation in SD-induced spatial memory impairment and suppression of neuronal cells proliferation and differentiation. The study suggested that microglia activation could be significant for memory impairment and targeting the same may provide an effective countermeasure against SD-induced neuroinflammation and spatial memory impairment.

## Additional files

Additional file 1: Figure S1. Sleep deprivation induces physiological and behavioral changes. A Track plot of training session and parameters. B Latency. C Path length. D Path efficiency. Probe test parameters. E Latency. F Path length. G Path efficiency [with hidden platform]. H Number of entries. I Time spent [no hidden platform]. Changes in physiological parameters such as J body weight. K Food intake. *p < 0.05 when compared to control treated with vehicle. Parametric and non-parametric Student’s *t* test was applied for the test parameters as required. (TIFF 453 kb)

Additional file 2: Figure S2. Standardization of minocycline dose on behavioral and inflammatory cytokine levels during SD. A Minocycline administration at 5 mg/kg dose provided an improvement in body weight along with food intake in comparison with sleep-deprived rats. Changes in the behavior predicted by B latency. C Path length. D Path efficiency [hidden platform]. E Number of entries. F Time spent [no hidden platform]. Fold changes in the pro-inflammatory cytokines. G TNF-α. H IL-1β. I IL-6 and the anti-inflammatory cytokines in the plasma. J IL-4. K IL-10. *p < 0.05 when compared to control treated with vehicle. ^ϕ^ *p* < 0.05 when compared to sleep deprived treated with vehicle. One-way ANOVA with Bonferroni post hoc test was used for body weight, food intake, latency, path length to reach the platform, time spent in the target zone, cytokine levels, and Kruskal-Wallis with Dunn’s post hoc test was applied for path efficiency to reach the platform, number of entries in the target zone. (TIFF 693 kb)

Additional file 3: Figure S3. Minocycline treatment improves SD-induced changes in behavioral and inflammatory cytokine levels in plasma during SD. Training session parameters. A Latency. B Path length. C Path efficiency. Track plot of probe test and parameters. D Latency. E Path length. F Path efficiency [with hidden platform]. G Number of entries. H Time spent [no hidden platform]. Fold changes in the pro-inflammatory cytokines. I TNF-α. J IL-1β. K IL-6 and the anti-inflammatory cytokines in the plasma. L IL-4. M IL-10. ^μ^ *p* < 0.05 when compared to first day of training. *p < 0.05 when compared to control treated with vehicle. ^ϕ^ *p* < 0.05 when compared to sleep deprived treated with vehicle. One-way ANOVA with Bonferroni post hoc test was used for latency, path length to reach the platform, time spent in the target zone, cytokine levels, and Kruskal-Wallis with Dunn’s post hoc test was applied for path efficiency to reach the platform, number of entries in the target zone. (TIFF 528 kb)

Additional file 4: Figure S4. Minocycline treatment improves temozolomide-induced changes in behavioral and cytokine levels in plasma during SD. A Track plot of the training session and probe test. Training session parameters. B Latency. C Path length. D Path efficiency. Probe test parameters. E Latency. F Path length. G Path efficiency [with hidden platform]. H Number of entries. I Time spent [no hidden platform]. Fold changes in the pro-inflammatory cytokines. J TNF-α. K IL-1β. L IL-6 and the anti-inflammatory cytokines. M IL-4. N IL-10 in the plasma. ^μ^ *p* < 0.05 when compared to first day of training, ^α^ *p* < 0.05 when sleep deprived treated with TMZ compared to control treated with TMZ. ^β^ *p* < 0.05 when sleep deprived treated with TMZ and minocycline compared to sleep deprived treated with TMZ. One-way ANOVA with Bonferroni post hoc test was used for latency, path length to reach the platform, time spent in the target zone, cytokine levels, and Kruskal-Wallis with Dunn’s post hoc test was applied for path efficiency to reach the platform, number of entries in the target zone. (TIFF 617 kb)

## Abbreviations

BDNF: Brain-derived neurotrophic factor
BrdU: Bromodeoxyuridine
BSA: Bovine serum albumin
DAB: Diaminobenzidine
DCX: Doublecortin
ELISA: Enzyme-linked immunosorbent assay
GFAP: Glial fibrillary acidic protein
H_2_O_2_: Hydrogen peroxide
HRP: Horseradish peroxidase
i.p.: Intraperitoneal
Iba-1: Ionized calcium-binding adapter molecule I
IHC: Immunohistochemical
MWM: Morris water maze
NGS: Normal goat serum
PBS: Phosphate-buffered saline
PFA: Paraformaldehyde
SD: Sleep deprivation
SGZ: Subgranular zone
SRSs: Sleep regulatory substances
SVZ: Subventricular zone
TMZ: Temozolomide
